# Exercise or Dietotherapy Is Not Better than Returning to a Regular Diet to Rebuild Lipid Homeostasis of Rats

**DOI:** 10.1155/2021/3047437

**Published:** 2021-10-01

**Authors:** Yuan Yang, Nan-Jun Xu, Jia-Hui Li, Ling-Feng Zeng, Gui-Hong Liang, Feng Zhang, Ming-Hui Luo, Jian-Ke Pan, He-Tao Huang, Yan-Hong Han, Jin-Long Zhao, Xiao Xiao, Chunlian Ma, Hua Liu, Yi Yang, Wei-Yi Yang, Jun Liu

**Affiliations:** ^1^The Second Affiliated Hospital of Guangzhou University of Chinese Medicine (Guangdong Provincial Hospital of Chinese Medicine), Guangzhou, China; ^2^Bone and Joint Research Team of Degeneration and Injury, Guangdong Provincial Academy of Chinese Medical Sciences, Guangzhou, China; ^3^The Second Clinical College of Guangzhou University of Chinese Medicine, Guangzhou, China; ^4^College of Health Science, Wuhan Sports University, Wuhan, China

## Abstract

Our aim was to explore the effects of dietary and behavior interventions on lipometabolism caused by an unhealthy high-fat diet and the best method to rebuild lipid homeostasis of this lifestyle. Apart from normal diet rats, 34 rats were fed with high-fat emulsion for 4 weeks and then intervened for another 4 weeks. Eight of them were classified into high-fat control group, and 9 were sorted into high-fat diet with rice vinegar group. Meanwhile, 10 were put into high-fat diet in swimming group, and 7 were just for refeeding normal diet group. Then, the data of body weight was recorded and analyzed. Indexes of serum samples were tested by kits. AMPK*α*, HNF1*α*, and CTRP6 in pancreas, liver, cardiac, and epididymis adipose tissues were detected by western blot. According to our experiments, swimming and refeeding groups reflected a better regulation on lipid homeostasis mainly by upregulating the expression of pancreas AMPK*α*. To be more specific, the refeeding rats showed lower T-CHO (*P* < 0.001) and LDL-C (*P* < 0.05), but higher weight gain (*P* < 0.001), insulin level (*P* < 0.01), and pancreas AMPK*α* (*P* < 0.01) than high-fat control rats. Compared with rats intervened by swimming or rice vinegar, they showed higher weight gain (*P* < 0.001), insulin level (*P* < 0.01), and HNF1*α*, but lower of CTRP6. In summary, refeeding diet functioned better in regulating the lipometabolic level after high-fat diet. Whatever approach mentioned above we adopted to intervene, the best policy to keep the balance of lipid homeostasis is to maintain a healthy diet.

## 1. Introduction

High-fat diet is the main cause of abnormal lipometabolism, such as hyperlipidemia, obesity, and cardiovascular disease. It is likely to be followed by unstable insulin levels, imbalanced energy metabolism, and depraved dyslipidemia [1]. Regulating the balance of lipid intake and exclusion is essential to maintain lipid metabolism. Excessive intake of lipids from diet affects the flux of substrates through lipogenesis and lipid oxidation to intervene related metabolism and insulin biological function [2]. In order to elaborate the mechanisms of disordered lipid metabolism, different high-fat diet rat models have been investigated by studies. For example, rats fed with a high-fat diet for 7 weeks were diagnosed with obvious hyperlipidemia and fatty liver [3]; 8 weeks of high-fat diet might lead to significantly increased body weight and lipid and glucose abnormalities in the rat models of hyperlipidemia and hyperglycemia [4]. In brief, disordered lipid metabolism caused by high-fat diet intervention is one of the classical methods in the metabolic field.

Since abnormal lipometabolism tends to develop into chronic refractory diseases with multitissues and organs, superior methods should be remarked as long-term and progressive effects. At present, studies have shed light on the potential lipid-lowering properties by some certain ways, e.g., swimming [5] and dietotherapy (e.g., rice vinegar) [6, 7]. However, these efficacious measures with quantitative standards may not be suitable for individuals to practice. As reducing lipid intake is the other way to regulate the imbalanced metabolism, low-fat diet and ketogenic diet are also heatedly discussed among the general diet modes [8, 9]. Here, we hypothesize that refeeding diet, an acceptable diet for returning to normal diet from high-fat dietary conditions, can also result in lowering lipid in certain ways (Figure 1).

As increasing evidence shows, AMP-activated protein kinase (AMPK) has emerged as an attractive target sensor to modulate lipid abnormalities and maintain energy homeostasis [10]. The strategy related to AMPK pathway on the regulation of whole-body lipid metabolism has been of interest, especially with the higher effect of heart, liver, and gonadal adipose tissue as compared with skeletal muscle by AMPK [11]. Moreover, liver and peripheral fat are important insulin-targeted tissues which can reflect the global lipometabolic level. Here, we focused on the related AMPK substrates: C1q/TNF-associated protein (CTRP) and hepatocyte nuclear factor-1 *α* (HNF1*α*). To reveal the best way to regulate lipometabolism by refeeding diet, rice vinegar, or swimming, the lipometabolism-related AMPK*α* in pancreas, liver, and cardiac tissues of high-fat diet rats was observed. The regulation of AMPK/CTRP6 and AMPK/HNF1*α* on fatty acid metabolism specifically in peripheral and liver tissues was also analyzed. Our ultimate goal is to explore the best lipid-lowering way to cope with abnormal lipometabolism problems and to provide a more scientific theoretical basis for a healthier dietary lifestyle finally.

This text has been preprinted in bioRxiv (https://www.biorxiv.org/content/10.1101/2020.01.08.899419v1).

## 2. Materials and Methods

### 2.1. Materials

#### 2.1.1. Ethics

All animal experimental protocols in the study were reviewed and approved by the Institutional Animal Care and Use committee of Wuhan Sports University. They were carried out under the guidelines of the National Institutes of Health Guide for the Care and Use of Laboratory Animals.

#### 2.1.2. Animals

39 SPF male Sprague-Dawley rats aged 2 months with the weight 200 ± 15 g was studied. These rats were purchased from the Research Center of Laboratory Animal in Hubei Province (No. 42000600014140). They were housed individually in stainless steel cages under controlled conditions for 1-week adjustment and then incorporated into our experiment. Apart from the normal diet group (NC, *n* = 5), other rats were fed with high-fat emulsion for 4 weeks and intervened by different methods for the following 4 weeks including high-fat control group (HC, *n* = 8), high-fat diet with rice vinegar group (HV, *n* = 9), high-fat diet with swimming group (HS, *n* = 10), and refeeding normal diet group (RH, *n* = 7). All rats were fed and kept in the clean SPF animal lab to ensure the experimental research was not affected by various factors. In addition, we observed and recorded the rats' spirit, diet, agility, defecation, hair, and color daily.

#### 2.1.3. Reagents and Equipment

Most reagents for SDS-PAGE and Oil Red O staining were purchased from Amresco or Biyuntian Bio of Shanghai. Others were listed as follows: HDL-C/LDL-C/TG/T-CHO test kit (Jiancheng Bio, Nanjing), Rat insulin ELISA kit (Huamei Bio, Wuhan), Rabbit anti-CTRP6 (Boosen Bio, Beijing), Rabbit anti-rat AMPK*α* (Emijie, Wuhan), Electrothermal thermostat incubator (Yuejin Medical, Shanghai), Vortex oscillator (Zhongxi Yuanda, Beijing), Multifunctional enzyme Standard instrument (Thermo Fisher, China), Centrifuge (Auchuangye, Beijing), Constant temperature culture oscillator (Zhicheng, Shanghai), Organization grinder (Jingxin, Shanghai), Ultrasonic cell crusher (Xinzhi Bio, Ningbo), Electrometer/Vertical electrophoresis bath (Liuyi, Beijing), Horizontal Shaker (Qilinbeier, Jiangsu), and BX53 Biomicroscopy (Olympus, Beijing).

### 2.2. Methodology

This text has been preprinted in bioRxiv (https://www.biorxiv.org/content/10.1101/2020.01.08.899419v1).

#### 2.2.1. Diet Protocol

After adaptive feeding, rats from HC, HS, HV, and RH in the first 4 weeks were given intragastric administration of 5 ml/kg high-fat emulsion daily [12]. In the following 4 weeks, rats from HC, HS, and HV were stilled taken with high-fat emulsion, and rats from HC and RH were returning to normal diet. In addition, rats from HV were taken with rice vinegar (10 ml/kg, daily) [13] for the following 4 weeks. High-fat emulsion included 20 g of lard, 2 g of cholesterol, 2 g of Sodium Cholate, 20 ml of Tween 80, 20 ml of Propylene Glycol, and 1 g of Propylthiouracil [14]. Rice vinegar of 9 degrees was diluted into 3 degrees and stored in the refrigerator.

#### 2.2.2. Exercise Protocol

Our exercise protocol was followed by the previous research of aerobic exercise for reducing animal stress and promoting health [15]. Only one group member of our research was responsible for the animal management and intervention on the rats of the HS group to avoid personality error. We adopted a moderate exercise protocol by 60 min swimming for 4 weeks (7 times/week) on average [16]. These rats underwent physical training within tepid water (30 ± 2°C) in experimental swimming pools (36 cm of depth).

Body weights of each rat were measured and recorded weekly throughout the experiment for further analysis. After 4 weeks of intervention, the rats were anesthetized with weight-adjusted injection of 1% sodium pentobarbital (4 ml/kg) followed by 16 h of fasting and inactivity. Thoracic blood was collected and used to get the serum which was stored at -20°C for the determination of metabolite concentrations. The adipose tissue samples (5 mm × 5 mm × 20 mm) of epididymis were quickly dissected in liquid nitrogen, then transferred to -20°C refrigerator for 30 min, and reserved for frozen tissue slices. The liver, pancreas, and epididymal fat tissues were quickly collected and snapped frozen in liquid nitrogen and stored at -80°C.

#### 2.2.3. Histological Analysis/Enzyme Assay/Western Blot

① Epididymis fat tissues were carefully dissected and placed on a cork with oxytetracycline. These fragments were cut into 5~10 *μ*m thick and covered with sliders, which were dried within 60 min at room temperature and then fixed in cold 10% formalin for 10 min. Then, the slides were rinsed immediately with distilled water, soaked in 60% of isopropanol, and stained with Oil Red O solution for 10 min. After separated with 60% of isopropyl alcohol until the background was colorless, the slides were washed again and stained with Mayer hematoxylin and then blued and distilled for several minutes. Finally, epididymis adipose slides were sealed and analyzed to get results of the degeneration and other changes of them. ② Analyses of metabolite concentrations (total cholesterol (T-CHO), triacylglycerol (TG), and cholesterol fraction (LDL-C/HDL-C) and insulin) were determined by enzymatic commercial kits followed by the manufacturer's instructions. The test methods of T-CHO and TG in rat serum were the same, which directly determined by the single reagent COD-PAP method according to the kit. Serum LDL-C and HDL-C were directly detected by the method according to the kit instructions. The content of insulin in serum was detected by the ELISA method according to the manufacturer's instructions. The main steps of these indexes above were to add buffer, sample, and reaction solutions with different concentration gradients in turn, to measure the OD value at different wavelengths, and to calculate the corresponding index concentration according to the formula for analyzing the content of serum samples. Samples from one experiment were running on the same plate in duplicate. And the average coefficient of variation was <10%. ③ The expressions of AMPK*α* (in pancreas, cardiac, and liver tissues), HNF1*α* (in liver), and CTRP6 (in epididymis adipose) were detected by protein immunoblotting. Samples were homogenized on ice with Organization grinder and Ultrasonic cell crusher (speed 10, 5 × 3 sec pulses) in RIPA buffer (ratio ~1 : 40), supplemented with protease and phosphatase inhibitors, and then centrifuged at 4°C (15 min with 12,000 rpm). The collected supernatant was used to determine protein content by a bicinchoninic acid assay. These protein samples, 10~20 *μ*g of protein, were prepared in loading buffer (ratio 1 : 1) and separated by electrophoresis on 10% SDS-PAGE gels (45 V, 45 min and 85 V, 90 min). Proteins were wet transferred onto nitrocellulose membranes at 350 mA with 2 h. Membranes were shaken in blocking buffer prepared with 5% nonfat dry milk in Tris-buffered saline/0.1% Tween 20 (TBST) for 1 h and then coming to the process of overnight incubation at 4°C with the primary antibody (dissolved in blocking buffer with 1 : 1000). Following primary incubation, the membranes were rinsed with TBST and incubated with horseradish peroxidase-conjugated secondary antibodies (dissolved to 1 : 10000) for 1 h at room temperature. Finally, signals were detected by enhanced chemiluminescence and subsequently quantified by densitometry and analyzed by the Image J software. The proteins expressed by the ratio of gray value of protein bands were normalized to *β*-actin.

#### 2.2.4. Statistical Analysis

The measured data were analyzed and processed by Spss19.0, GraphPad prism5, Image-pro plus 6.0, and CurveExpert1.3. Comparisons between different groups were made using unpaired, two-tailed *t*-tests. Body weight of different groups over time was determined using a one-way ANOVA followed by Tukey's post hoc analysis. The data analyzed were expressed as mean ± SE, *P* < 0.05 indicated statistical difference, *P* < 0.01 indicated that each data had significant difference, and *P* < 0.001 indicated an extremely significant difference.

## 3. Results

### 3.1. Body Weight Changes by High-Fat Diet and Different Interventions

The analysis of body weight changes of two experimental periods (1~5 week and 5~9 week) was taken from a weekly statistic protocol (Table 1). In Figure 2(a), an upward trend of increase in the weight of rats was noticed in the first 4 weeks, while statistic differences did not become obvious until the following four weeks. Combined with Figure 2(b), except for the consistently increasing trend in the normal diet group and the refeeding group, the body weights of other three groups were decreasing distinctly. Specifically, the body weight gain of HC, HV, and HS rats during 5~9 weeks was significantly lower than that of other two groups (NC and RH) (*P* < 0.001) in Table 1. However, there was no difference among HC, HV, and HS groups, nor significantly difference on the body weight gain of RH and NC during 5~9 weeks. In brief, the weight of rats with refeeding diet kept increasing, while rats with high-fat diet that were also intervened with vinegar or swimming experienced weigh loss.

### 3.2. Morphological Changes of Adipose Tissue with Oil Red O Staining

The OD value of Oil Red O of different groups showed different histological changes on epididymis adipose (Table 1). Compared with NC, the OD value of HC and HV tended to be lower (*P* < 0.05), but that of RH was higher (*P* < 0.05). Compared with HC, higher OD value was shown in HS (*P* < 0.05) and RH (*P* < 0.01), but the OD value of RH was even higher than HS (*P* < 0.05). According to S-Fig, normal lipid droplet in HC was not obvious among the high-fat diet rats, and most of them were partial flakes with diffuse steatosis. The HV group showed similar scattered lipid droplets as HC did, while it showed a lower degree of steatosis, and some irregular red crystals could be ignored. Scattered lipid droplets were similar in HC and HV, and the latter demonstrated a lower degree of steatosis. And some irregular red crystals could be ignored. There were also variations of steatosis in HS and RH, and the lipid droplets in these groups were more obvious than those of HC. The fat depot in RH was less punctate with little steatosis, while the amount of lipid droplets in the tissue was higher than that in HV and HS. Compared with other interventions, the HS group showed similar normal lipid tissue in Oil Red O with NC, which means swimming was better to alleviate pathological adipose changes on high-fat diet rats.

### 3.3. Serum Lipid and Insulin Levels in Blood

#### 3.3.1. Serum Lipid Levels

As shown in Figure 2(c), the indexes of serum lipids (T-CHO, TG, LDL-C, and HDL-C) in these groups were different, among which T-CHO was most obvious distinctly, TG and LDL-C were individual different, and HDL-C had no statistical difference. According to Table 1, compared with NC, it was higher of T-CHO concentration in HC (*P* < 0.001) and HV (*P* < 0.01) and higher of LDL-C concentration in HC (*P* < 0.05). Compared with HC, HS was significantly lower in TG (*P* < 0.05), and RH was significantly lower in T-CHO (*P* < 0.001) and LDL-C (*P* < 0.05). Compared with RH, there was a significant higher of T-CHO concentration in HV (*P* < 0.01) and HS (*P* < 0.05). Therefore, swimming could specifically reduce TG concentration. And refeeding diet could specifically reduce both T-CHO and LDL-C, while rice vinegar had no significant effect on improving blood lipid metabolism.

#### 3.3.2. Serum Insulin Levels

It was shown a significant difference in insulin levels among the groups in Figure 2(d). Compared with NC, lower serum insulin level was observed significant in HC, HV, and HS (*P* < 0.001) in Table 1, while there was no difference among these 3 groups. Specifically, the insulin levels in RH, which was higher than HC, HV, and HS (*P* < 0.01), did not show a significant difference compared with NC. That is, the insulin level in high-fat diet rats was lower. It could be reversed by refeeding, rather than swimming or rice vinegar.

### 3.4. Expression of AMPK*α* in Pancreas, Liver, and Cardiac Tissues

As shown in Figure 3(a), A, AMPK*α* expression in the pancreas of each group was significantly different. The expression in rice vinegar, swimming, and refeeding groups was significantly higher than that of other groups (*P* < 0.001). It was even higher in the HS group than that in the RH group (*P* < 0.001). AMPK*α* expression of liver shown in Figure 3(a), B indicated that there was no distinct difference among these groups, while different interventions did affect liver AMPK*α* which was higher in RH (*P* > 0.05) and lower in HC (*P* > 0.05). As shown in Figure 3(a), C, compared with the NC group, cardiac AMPK*α* expression in each group increased after high-fat diet, and the expression was significantly higher in the HV group (*P* < 0.01) and the swimming group (*P* < 0.001). Therefore, different interventions had distinct effects on the expression of AMPK*α* in special tissues. Both swimming and rice vinegar had impacts on pancreas and cardiac tissues, while more obvious influence was shown on the HS group. The refeeding group had a significant effect on the pancreas. The sign of its influence on liver tissue was spotted but no statistic difference was shown by far.

According to the results above that AMPK*α* expression in pancreas was higher after different interventions, we analyzed the relationship between pancreas and lipometabolism furtherly. The correlation between pancreas AMPK*α* and blood lipids was discussed subsequently by Pearson analysis in S-Tab. 1. It turned out that, among all lipid metabolite concentrations, only TG was found to be linked to pancreatic AMPK*α* (*P* < 0.05). That is, swimming could specifically reduce the TG concentration in blood lipids and showed more effect on pancreas AMPK*α* than rice vinegar or refeeding did.

### 3.5. Expression of HNF1*α* and CTRP6 in Tissues

As shown in Figure 3(b), A and B, there was no significant difference between NC and other 4 groups (*P* > 0.05) on the expression of HNF1*α* in liver and CTRP6 in periepididymal adipose, nor the difference was found among HV, HS, and RH (*P* > 0.05), while various expression levels of HNF1*α* and CTRP6 in each group affected by different methods indicated distinct outcomes in Figure 3. Theoretically, effective interventions probably functioned with higher HNF1*α* levels and lower CTRP6 compared with HC. However, the results did not show obvious effects on high-fat diet rats with lower HNF1*α* expression by rice vinegar, swimming, or refeeding. In addition, except for RH, CTRP6 expression did not turn to be lower in HV or HS. A further analysis showed there was neither a significant relationship between liver HNF1*α* and AMPK*α* in different tissues nor a correlation among blood lipid, pancreas AMPK*α*, and CTRP6 protein in rats in S-Tab. 2 and S-Tab. 3.

## 4. Discussion

In this study, we demonstrated different interventions by rice vinegar, swimming, and refeeding to high-fat diet rats might lead to discrepant effects. The results of refeeding showed, although there was no function of losing weight in refeeding rats, the content of T-CHO and LDL-C, insulin level, and AMPK*α* expression in pancreas and liver tissues were regulated significantly. In general, in addition to the rice vinegar group, the interventions of swimming and refeeding did play an important role in regulating blood lipid metabolism. However, we also noticed that their effects on body weight and insulin level were completely opposite, and blood lipid composition was also different. The above conclusions provoke our further discussion: How do dyslipidemia, body weight, and insulin level work with each other? And what is the possible pathway related to AMPK*α* and lipid metabolic regulation in various tissues?

Previous studies demonstrated that weight gain was a main manifestation of dyslipidemia, especially on T-CHO, TG, and lipoproteins in serum lipids [17]. In our study, however, continuous high-fat diet had an effect on weight loss, which was even more obvious in rice vinegar and swimming groups. On the contrary, the rats of the RH group gained weight clearly, which was closer to normal diet rats and had significant function on regulating serum lipid and insulin levels. It gave us a second thought that body weight, although correlated with dyslipidemia, might not be used as a direct indicator to reflect the level of lipometabolism. Refeeding diet, superior to swimming or rice vinegar, significantly helped to regulate dyslipidemia specifically by lowering T-CHO and LDL-C in our experiment. They were consistent with the previous conclusion that the effect of diet was mainly lowering TG and LDL-C, and exercise was regulated predominantly by lowering fasting TG [18]. We also concluded that rats with high-fat diet showed a significant decrease of insulin level in serum, which increased more obviously in refeeding rats than that of other interventions. Thus, it was suggested that insulin level probably regulated dyslipidemia with balanced TG level, but whether it could restrict the content of TG continuously needs further study.

Studies on dietary restrictions have shown that altered meal patterns could be used to prevent certain metabolic diseases [19]. Our study reveals that refeeding with high-fat diet improves lipid homeostasis, which is seldom discussed by other researches. Specifically, the regained body weight and lower T-CHO and LDL-C by refeeding from high-fat diet was followed by significantly higher insulin levels, which is an important marker of regulating the lipometabolism globally. In addition, the fat depot in RH with less punctate steatosis means histological changes of lipid droplets were recovered partly by refeeding from high-fat diet. AMPK*α* expression of RH was significantly higher in pancreas and liver than high-fat diet rats. HNF1*α* is a typical protein of liver. The expression of it in RH was higher than that in HV or HS but still lower than HC. On the contrary, CTRP6 of periepididymal adipose in RH was closer to that in the normal diet group. The above results highlight the therapeutic potential of refeeding diet, independent of alterations in weight loss or other consumption, as a persuaded advice to ameliorate dyslipidemia changes in lipometabolic-associated pathology.

Our study showed a significantly higher AMPK*α* expression, particularly in pancreas among different tissues after intervening high-fat diet rats. And it showed a significant negative correlation between AMPK*α* in pancreatic and TG. It was discussed in our study that rats intervened only by swimming showed lower TG and higher expression of pancreas AMPK*α*. We got the hypothesis that swimming, rather than refeeding, could affect dyslipidemia by specifically moderating pancreas AMPK*α*. The intervention of refeeding showed a superior effect on liver AMPK*α* and insulin level than others. Probably, mechanisms of it on insulin level and lipometabolic disorders might be related to targeted tissues of insulin, i.e., liver and surrounding adipose. Deficiency of HNF1*α* in liver lipometabolism may lead to diabetes and hypercholesterolemia by increasing bile acid and cholesterol synthesis [20]. The cross-talking of insulin levels and AMPK*α*/HNF1*α* supports AMPK-mTOR-HNF1*α* pathway for the treatment of lipometabolism and insulin dysfunction [21]. However, HNF1*α* expression in RH did not show lower than that in HC, which means the effect on dyslipidemia by refeeding might not work through AMPK-mTOR-HNF1*α* signal pathway. CTRP6 contains a globular domain which inhibits to mediate the phosphorylation and activation of muscular AMPK. Our study showed the expression of CTRP6 in adipose tissue was only decreased in refeeding rats, and its effect on lowering lipid may relate to liver AMPK*α* and periepididymal adipose CTRP6. Combined with significant changes of T-CHO in serum lipid and insulin levels, the peripheral regulation of lipometabolism by refeeding probably mediates targets from liver to periepididymal. We will focus on AMPK-ACC-CTRP6 signal pathway for further research on this regulation in subsequent experiments.

In the process of this experiment, there are some defects as the following: Analysis of food intake should be added in the experiment, or the rats should be given a fixed diet intake to be compared among different groups; the decline in lowering lipid was accompanied by peripherally regulating AMPK*α*, CTRP6, and insulin levels.

In summary, refeeding and swimming significantly regulate lipometabolic after high-fat diet through indicators of different target organs, such as AMPK*α* in pancreas, liver, and cardiac tissues. Refeeding diet, compared with other interventions, functioned better in regulating the lipometabolic level after high-fat diet. Whatever approaches we adopted to intervene, the best policy to keep the balance of lipid homeostasis is to maintain a regular diet.

## Figures and Tables

**Figure 1:** Balance of blood lipid metabolism and corresponding interventions. Exogenous and endogenous lipids maintain blood lipid levels. Excessive fat intake needs to accelerate the metabolism and limit the synthetic lipids in vivo to restore the balance of blood lipids. The process involves the coordination of multiple organs: ① excessive fatty acids (FA) in adipose tissue need to be metabolized through the liver and bile, ② reducing insulin-mediated glucide (Glu) converses to excessive TG, and ③ reducing the synthesis of TG and T-CHO in liver. Excessive T-CHO will come to the heart from blood circulation and cause serious cardiovascular diseases. There are two ways to regulate the abnormal lipid metabolism. One is a therapeutic diet that blocks dyslipidemia from exogenous sources. The other way is to exert biological effects on the corresponding pathway and regulate lipid metabolism in vivo by exercise, drugs, functional supplements, and so on.

**Figure 2:** Weight and blood analysis. Values are means ± SE; compared with NC, ^#^*P* < 0.05 and *^###^P* < 0.001; compared with HC, ^※^*P* < 0.05 and ^※※※^*P* < 0.001; compared with RH, ^∗^*P* < 0.05 and ^∗∗∗^*P* < 0.001; (a, b) note that 0~1 w indicated the weight of rats fed adaptively for 1 week with no significant body weight changing among different groups, 1~5 w indicated the weight of rats on a normal/high-fat diet for 4 weeks, and 5~9 w indicated the weight of rats with different interventions for the following 4 weeks.

**Figure 3:** (a) Relative expression of AMPK*α* in pancreas, liver, and cardiac tissues. (A) The relative expression of AMPK*α* in pancreas, (B) the relative expression of AMPK*α* in liver, and (C) the relative expression of AMPK*α* in cardiac tissues. (b) Relative expression of HNF1*α* in liver and CTRP6 in periepididymal adipose. (A) The relative expression in liver and (B) the relative expression of CTRP6 in periepididymal adipose. Values are means ± SE; *n*: No. of rats. Compared with NC, ^#^*P* < 0.05 and *^###^P* < 0.001; compared with HC, ^※^*P* < 0.05 and ^※※※^*P* < 0.001; compared with RH, ^∗^*P* < 0.05 and ^∗∗∗^*P* < 0.001.

**Table 1:** Changes in body weight, lipid metabolite concentrations, and OD value of Oil Red O on epididymis adipose of rats.

	NC (*n* = 5)	HC (*n* = 8)	HV (*n* = 9)	HS (*n* = 10)	RH (*n* = 7)
BW gain (g)/1~5 weeks	80.4 ± 31	56.8 ± 13.72	60.8 ± 21.16	62.6 ± 21.52	26.6 ± 25.7^#^
BW gain (g)/5~9 weeks	49.4 ± 57.46	-40.2 ± 27.97^###^	-81 ± 33.77^###^^∗∗∗^	−57 ± 8.8^###^^∗∗∗^	36.5 ± 15.07^※※※^
T-CHO (mg/dl)	2.86 ± 0.37	5.40 ± 0.41^###^	4.65 ± 2.02^##^^∗∗^	4.23 ± 1.05^∗^	2.66 ± 0.96^※※※^
TG (mg/dl)	3.29 ± 0.63	3.65 ± 1.34	2.45 ± 1.37	2.27 ± 0.92^※^	3.56 ± 0.83
LDL-C (mg/dl)	0.44 ± 0.41	1.21 ± 0.64^#^	0.59 ± 0.46	0.91 ± 0.55	0.37 ± 0.33^※^
HDL-C (mg/dl)	0.58 ± 0.43	0.86 ± 0.58	1.48 ± 1.26	0.78 ± 0.46	0.56 ± 0.42
Insulin (nIU/ml)	200.8 ± 61.48	57.29 ± 34.32^###^	48.40 ± 22.74^###^^∗∗^	48.56 ± 15.15^###^^∗∗^	157.29 ± 34.63^※※^
OD value	0.3337 ± 0.0398	0.2479 ± 0.0103^#^	0.2483 ± 0.0197^#^^∗∗^	0.3059 ± 0.0334^※^^∗^	0.4533 ± 0.0457^#※※^

Values are means ± SE; *n*: No. of rats; BW: body weight; T-CHO: total cholesterol; TG: triacylglycerol; LDL-C/HDL-C: cholesterol fractions; OD value: the OD value of Oil Red O on epididymis adipose. Compared with NC, ^#^*P* < 0.05 and ^###^*P* < 0.001; compared with HC, ^※^*P* < 0.05 and ^※※※^*P* < 0.001; compared with RH, ^∗^*P* < 0.05 and ^∗∗∗^*P* < 0.001.

## Data Availability

All data generated or analyzed during this study are included in this published article.

## Supplementary Materials

Supplementary Materials The results of correlation coefficients among blood lipid, pancreas AMPK*α*, and periepididymal adipose CTRP6 in rats are listed in S-Tab.1/2/3. Oil Red O staining in epididymis fat tissues of rats is shown in S-Fig.
